RETRACTED

# “Crisis Within the Walls”: Rise of Intimate Partner Violence During the Pandemic, Indian Perspectives

**DOI:** 10.3389/fgwh.2021.614310

**Published:** 2021-05-28

**Authors:** Vasundharaa S. Nair, Debanjan Banerjee

**Affiliations:** ^1^Department of Psychiatric Social Work, National Institute of Mental Health and Neurosciences, Bengaluru, India; ^2^Department of Psychiatry, National Institute of Mental Health and Neurosciences, Bengaluru, India

**Keywords:** COVID-19, pandemic, domestic abuse, intimate partner violence, women

## Abstract

The ongoing coronavirus disease 2019 pandemic has been a social “un-equalizer,” besides being a global health threat. Gender inequality has been globally prominent during the outbreak and the consequent lockdown. Although domestic abuse and intimate partner violence have increased due to chronic entrapment, overcrowding in families, enhanced substance use, distorted relationship dynamics, travel restrictions, and reduced healthcare access, coercive sexual practices have also been on the rise. In low- and middle-income countries, the lack of awareness, societal pressure, administrative apathy, fear of legal hassles, and inadequate knowledge–attitude–practice related to help-seeking lead to underreporting and mismanagement of domestic abuse, which can perpetuate its vicious cycle during the ongoing crisis. India, with its socio-culturally diverse population, has been one of the nations worst hit by the pandemic. With the rise in reports of gender-based violence on the premise of preexisting gender inequality and minority stress, concerns behind “closed doors” are as threatening as the infection itself. With this background, the authors highlight the backdrop of domestic violence as a “hidden pandemic” during the coronavirus disease 2019 crisis, drawing on perspectives from India and briefly reviewing the data from other nations. The role of mental health education and digital literacy as mitigating strategies is subsequently discussed.

## PROLOG

“Injustice anywhere is a threat to justice everywhere.”

(Dr. Martin Luther King Jr., 1963) (1).

Coronavirus disease 2019 (COVID-19) has been a worldwide medical issue. Beyond just the purview of public health, it has affected the daily lives of billions, either isolating them in detachment or abandoning them with their families for significant stretches more than ever (2). The negative social outcomes are steadily getting evident, as “human conduct” can change uniquely under emergency and “inside shut dividers.” One of the offshoots is the worldwide “evil” of domestic violence, which has expanded particularly. It incorporates sex-based brutality, child and elderly maltreatment, and intimate partner violence (IPV). The contributing components during this pandemic are expanded pressure, travel limitations forced by lockdown, expanded conjugal friction, uncommon staying periods with the accomplices, stuffing, stress, nervousness, money-related emergency, and substance misuse (3).

RETRACTED

Further intensifying the articulation of the situation are the elements of underreporting, poor accessibility to social and medical care, domestic dangers, and absence of mindfulness and sensitivity even among health care professionals. Families with prior maladaptive treatment make it an increased “norm,” legitimized by the disconnection and lockdown. With the expansion in the number of days in the lockdown, reports of the increased number of cases of IPV were known to the entire world. The United Nations (UN) defines IPV as any behavior by an intimate partner or ex-partner who causes physical, sexual, or psychological harm, including physical aggression, sexual coercion, psychological abuse, and controlling attitudes. It is often viewed inseparably from domestic violence or abuse. Specifically, when directed toward the female sex, it can be intimidation, animosity, or arbitrary deprivation of autonomy, all of which have detrimental effects on their overall being and quality of life^1^. The UN Secretary-General Antonio Guterres called out for a “ceasefire” on April 6, 2020, to address the “horrific global surge in intimate partner violence” ^1^. In an effort to focus on public health strategies during the pandemic, the suffering of this vulnerable group has only intensified. For this article, we will be using IPV and domestic violence interchangeably. IPV has been a well-established risk factor and considered a social evil for women through decades (4) with far-reaching socioeconomic and public health consequences (5). However, with the “stay-home directives,” the last year of a pandemic has seen an unprecedented and chronic rise in this traumatic experience (6). Factors such as chronic entrapment with families, increased substance abuse, overcrowding, unemployment, isolation, loss of income, poverty, anxiety, and stress, all have led to disproportionately increased risk in women and children (7). It is important to understand that IPV can further exacerbate human rights crises and social injustice that fracture resilience and psychological health, which are crucial attributes during a crisis such as COVID-19.

Violence and disasters have an established correlation. The eruption of Mount St. Helens in 1980, Hurricane Katrina in 2005, the Black Saturday bushfire, 2009, and the Earthquake in Haiti, 2017 are classic examples of IPV that were established in the background of family stressors, reported aggression, unemployment, and other associated stressors (8). Studies have demonstrated a 98% increase in “physical victimization” of women in the post-Katrina aftermath (9). Similar spikes have been seen after the tsunami and Indian Ocean earthquake of 2004 (10), as well as the Black Sunday Australian bushfires (11). It has been hypothesized that preexisting social and ecological issues are further destabilized by the disaster-related uncertainty, stress, displacement, fear, disruption of social infrastructure, and economic downfall that lead to the vicious cycle of evils such as domestic violence (12). Even previous outbreaks such as Ebola, cholera, Zika, and recently Nipah have led to disruptions in familial relationships and increased domestic violence (13). Although the statistics are yet rising systematically on the international platform, the gender-based violence rates are increasing in the United Kingdom (UK) National Domestic Abuse Helpline (14). A similar rise has also been seen in other countries heavily affected, such as Spain, Italy, and China (15). It is vital to recall that persistent domestic abuse can have to impede psychosocial and physical outcomes, and it has already been understood as a “social evil” that will be tough to identify and tackle. This paper thus plans to spotlight this concerning aspect of the pandemic and highlights some of the psychosocial factors that may prompt this issue from the Indian context. The role of mental health education and its integration into general well-being as a measure of mitigation are examined in the end.

RETRACTED

## Problem Premise

“I am extremely tired all the time. I am no longer in the mood to explain as to how work from home is an equally taxing thing. I have to manage my home, my children, and everything in my office. This is so new, I am so done with this routine. I wish for the day I will sleep peacefully and also someone who would just listen, if not completely understand at least try to understand…”

**(A software engineer from Bangalore, on working from home during the lockdown)**.

“The government is stating that they have done this lockdown for the betterment of the country but here I am finding it difficult to deal with my husband. His usage has increased and I have n place to run to or go to. I can't call at my house as he keeps checking me and what all am I doing. If by any chance I even dare to answer back or refuse, all the anger is on me, I will be beaten up and I know I have no choice either. Rather than dealing with this torture, I would prefer to die of Corona.”

**(A crisis call to our helpline, from a lady staying with husband in rural Karnataka)**.

RETRACTED

(**Both excerpts are altered to some extent for anonymity and obtained with informed consent. They have been added to provide a real-life perspective to this article).

**The excerpts earlier might be from different poles of social class but mirror a common theme: the lack of understanding of close family members, altered perceptions about women's independence, and substance abuse, all eventually contributing to domestic violence**.

Worldwide, one-third of women experience physical or sexual violence during their lifetime. At least two in five individuals in relationships experience some form of violence by partners (16). The intent is not to focus that domestic abuse is directed only on women; however, in most cases, they are the victims, and this comparable point of view will be maintained throughout this article. Violence against women is, in fact, on the rise, especially in developing and populous countries such as India. India has been disreputable for gender-based violence, ranked as the fourth country in the world for gender inequality, according to public perceptions (17). As per the National Crime Research Bureau data, nearly 90,000 cases related to crimes against women were registered against women in 2018, higher than 86,000 in the previous year^2^. Nearly 33% of these were some form of domestic abuse. The National Family Health Survey-4 of 2015–16 reported that more than three in 10 Indian women between 15 and 49 years had experienced physical violence in relationships, with 85% of cases the perpetrators being their male partners (18). These certainly speak to hint of something larger, as social shame, dread, and legitimate issues forestall revealing of most cases. As billions have been stranded at their homes for “social distancing” trying to control the episode, domestic violence has been rising. The National Commission of Women in India received 239 complaints between March 23 and April 16, as compared with the previous lockdown phase having 123 cases (19). A large number of these were homegrown in nature, related to bigamy, polygamy, dowry-related issues, substance abuse, and marital disharmony. It is also important to understand that not all forms of domestic abuse are physical violence: restriction of rights, mobility, autonomy, and sexual harassment are also equally traumatic. Mental and money-related maltreatment may be ongoing and subtle but eventually normalized, although having a more prominent effect over the long haul. Furthermore, controlling behaviors, gender-based stereotypes, gender discrimination, misogynistic attitudes, and jealousy can increase during a disaster crisis that reinforces domestic violence (11).

RETRACTED

To date, most of the data related to IPV come from the developed nations. Hubei in China, which formed the epicenter of COVID-19, reported a tripling of domestic violence in February 2020 as compared with that of last year, based on police reports (20). After the first month of the stay-at-home orders, a 20–30% increase in domestic violence calls was reported in the nine United States (US) metropolitan cities (21). However, subsequent data from the IPV helplines were mixed, and it can be possible that fear, physical proximity to the abusive partners, and travel restrictions impacted the reporting (6). The US has mentioned IPV as a “hidden pandemic” in the background of COVID-19, and domestic violence calls for service to the police increased by 7.5% from March to May 2020, at the initiation of lockdown (22). This increase was at a maximum (9.7%) in the first few weeks when social distancing measures started. Households with a preexisting history of discord, substance abuse, IPV, and litigations related to the same showed a significant increase. Initial reports from the National Domestic Abuse helpline (UK support services) showed an increase in service use, which was consistent with similar patterns in Spain, France, and China (23). Toward the end of the last year, Boserup et al. (24) highlighted “alarming trends in US domestic violence” during the pandemic crisis in various areas of Portland, San Antonio, and Jefferson County, Alabama. The increase in police reports ranged from 10 to 27%. The UN Women (25) reported an increase of 30% in domestic violence documentations in France since the initiation of lockdown. A similar increase in the incidence of IPV has also been reported in Argentina, Singapore, and Cyprus. However, most of these data are anecdotal and based on individual reports, which bring in bias and impact its reliability. In one of the largest studies, an online survey of 15,000 women from Australia conducted in May 2020 revealed that 4.6% of the participants experienced sexual or physical violence from their partner. Whereas, 5.8% experienced coercion and control, 11.6% reported facing at least one form of harassment, controlling, or emotionally abusive behavior (26). The violence had escalated in 3 months preceding the survey, and nearly all the participants who faced abuse reported individual and social barriers in help-seeking.

Understand that each rule of the government for the advancement of the communities accompanies the part of comorbid psychological and psychosocial difficulties, which then have a straight correlation with the quality of life and mental health of the individuals. The helpline services working across the country have received close to a hundred calls reporting “physical, emotional, and verbal abuse” (27). Urgent steps of spreading awareness, mass sensitization, community-based approaches, and active inclusion of women and child safety measures during this crisis are needed to fight this “social wickedness.” Although the Prevention of Domestic Violence Act exists in India, very few are aware of the legal provisions available, and hence, underreporting is the norm rather than the exception (28).

RETRACTED

## Domestic Abuse: The Vicious Cycle

Understand that savagery happens regardless of gender, class, caste, creed, time, or place. Family, considered as the primary support system, becomes the primary site of abuse and brutality. Sociologically, role allocation being chauvinist in nature has brought about the division of household work as “women's work.” The change in the daily home routine and structure due to the increased amount of time spent by different individuals altogether increases the role strain and affects the ambiance of the house. Family in this context has been often termed by individuals as a “primary site of exploitation,” and the same trend has been seen to rise with the increasing number of days in lockdown. Women over the helplines in the country have stated restrictions in terms of access, food, and non-provision of masks, thereby making them use “dupattas and pallus” for respiratory hygiene, non-access in the ration card, liquefied petroleum gas, and clinics. Most of the women in the country do not even have access to phones for communication, as they have to depend upon their husbands, fathers, or brothers. The ineffectiveness of the law wherein marital rape is still not considered a criminal act adds to the insult. All these factors have a holistic effect on the affected person's health and rights (29). Clearly, in times of monetary and financial recession, human behavior tends to be impulsive, reckless, controlling, and aggressive, and the brunt usually goes down the patriarchal power-hierarchy, so significant for India. Here are a few factors contributing to the endless loop of domestic abuse, especially during pandemics.

- *Lack of awareness on the availability of hotlines:* Most of the individuals, who undergo violence, cannot report it or notify the authorities due to the absence of knowledge about the hotlines. An increase in awareness and promotion will increase the help-seeking behavior and reporting among them. The penetration of these helplines in rural areas is a challenge.
- *Misinformation and role of social media:* For all pragmatic reasons, COVID-19 has turned into a digital “infodemic” with data overload adding to the stress burden. Various gossip-mongering and false news over social media appear as hindrances in the method of self-sufficiency for women, increasing fear of infection and transmission (30). Misunderstanding the precautions of a pandemic might alter social perceptions leading to faulty attitudes among partners.
- *Lack of health care access:* Many cases that are now enlisted at various social centers or hospitals might be lost to follow-up and review during COVID-19 due to the non-availability of many health services and travel limitations. These cuts off the vulnerable from social care and can perpetuate the already existing violence.
- *Lack of sexual and reproductive health services*: In the current condition, it has been hard for them to connect with the healthcare professionals who provide sexual and reproductive health services face to face and simultaneously; an equivalent has not been provided currently over helpline services either, making it difficult for them, thereby increasing the rate of unprotected sex, forced sex, pregnancy, and marital rape (31). The absence of thought on healthy sexuality and intimacy practices is prevalent during this pandemic, which often leads to sexual frustration and coercive and risky sexual interactions. Banerjee and Rao, in their detailed review on sexual well-being and intimacy during pandemics, highlight the possible rise of coercive and non-consensual sexual practices, sexual deviations, and increased marital disharmony during the ongoing crisis, all of which can contribute to gender-based stress and violence. The authors also mention “minority stress” as one of the factors promoting discrimination, stigma, and stereotyping among women as “passive recipients of sufferings” with reduced social support, disclosure, and help-seeking, thereby perpetuating the cycle of trauma and abuse (32).
- *Fear of the police/legal hassles and stigma:* Most women stay away or avoid reporting to the police out of fear, resistance, or the dread of exploitation by the police. They tend not to have gotten ahead and come and seek help, thereby increasing the difficulty. It cannot be generalized, as the same number are eager to help. Be that as it may, some awful encounters, as a rule, pollute the bigger situation. The social and self-stigma related to disclosure and normalization by the families further lead to underreporting.
- *Difficulty in managing family:* With numerous individuals living under the same roof, women in general deal with the tasks of the family as well as of the parts of childcare because of the conventional structures, role strain, and role allocation that may not adequately manage, thereby causing difficulty in the form of hostility and concern.
- *Objectification of women:* Objectification theory states that women are treated as an object to be valued for its use by others, and she is viewed as a physical object of a “male want.” This behavior in the Indian tradition is found as a “normalized heteronormative tradition,” thereby increasing the concerns of name-calling, self-objectification, several risks, and stressors, thereby affecting the physical and mental health of women (33). Motion pictures and media often add to this, worsening this conviction framework.
- *A cycle of violence:* Alcohol as a mood enhancer has a direct correlation with feelings of anger, frustration, and irritation. A man's impression of the need to consent to the gender norms could be exacerbated by substance abuse, thereby shifting the focus on women. This then results in violence. Due to the vulnerabilities of women, the endless loop might continue from the women to offsprings, a further force from the family of origin, the expected normalcy from the family of procreation, and difficulty in the accessibility and availability of the legal aid services add to the problems (34).
- *Lack of livelihood*: Women who are unable to go to work during this crisis have to critically balance “work from home” and “work for home.” Perceptions of the family might interfere with their work patterns with added domestic responsibilities, the clash of which leads to discord. Many might be in financial crisis, worsening their autonomy in their respective familial circles.
- *Knowledge–Attitude–Practice gap*: This is perhaps the most important contributing factor (35). For decades, domestic violence has been normalized by social strata across all classes, so much so that the awareness and need for prevention are undermined grossly. The effect of mental and physical well-being is also largely misinterpreted.

RETRACTED

## Mental Health Literacy: A Mediating Tool

The common dictum for all health professionals is that “you do not ask, and they do not tell.” In a busy clinical practice during a global public health crisis, time management and triaging are often vital issues that lead to unintentional missing of subtle signs of IPV. Irrespective of speciality, during this pandemic, the physicians and healthcare workers need to be sensitive to the exploitative relationships, crisis calls for help, marital discord, dealing with children witnessing IPV, and psychological manifestations such as anxiety, depression, post-traumatic stress, somatization, etc. (36). Krishnakumar and Verma (37), in a recent study, applied the routine activity theory framework for the content analysis of media reports related to domestic violence in India during the lockdown. The three components of the routine activity theory in criminology are motivated offender, the absence of a capable guardian, and a suitable target. Findings revealed alcohol and unemployment to be the “motivators.” The symbolic value assigned to women in society and easy accessibility made them the “targets,” whereas a shortage of police and travel restrictions made them vulnerable to IPV. The authors highlighted the need to integrate these measures into the public health system for IPV prevention. The role of mental health professionals and media is immense, and inter-sectoral collaboration with the policymakers and legal services is the key. Detailed recommendations for all levels of stakeholders to prevent IPV in India are highlighted by Krishnan et al. (28) and will not be repeated here. We will be focusing on the mental health education (MHE) approach. MHE is specially equipped at times of such crisis with strategies ranging from individual to systemic and community level in promoting mental and social well-being (38). Domestic abuse being an integral component of both, MHE can be basic to enable awareness and understanding in the communities and aid in the larger reach with the assistance of media and community health workers. It can also use technology for training and advocacy programs. Here are a few ways in which that can be brought about.

- *Increasing awareness:* Information–education–communication materials can be prepared to ensure the understanding of the people on IPV and the help-seeking behavior through helplines. Socioculturally appropriate and multilingual infographics can be simple aids to put out the message to the masses. Digital literacy needs to involve women of various socioeconomic and ethnic groups for greater community outreach and education. Both early identification and reporting of abuse should be encouraged among all individuals.
- *Boosting the manpower:* Although crisis management and psychosocial first aid are structured as a package by the mental health care professionals, the aspect of networking, collaborating, and ensuring capacity building among them could be done through the training of the police personnel and other individuals who volunteer and are ready to provide protective services.
- *Provision of Legal Aid work:* Statistics, once generated, could be shared with the police authorities, women cells, and legal aid cells wherein the immediate details could be planned, and also in case of urgency 24 × 7 legal aid courts, ambulance services could be set up.
- *Community outreach*: Local, state, and national government could be provided with sensitive and comprehensive messages in the form of audio, video, and written methods such that maximum message can be circulated and processed for the beneficiary. Tele-sessions can be immensely helpful for a wider outreach with the integration of all levels of healthcare.
- *Social stigma campaigns*: Involving all levels of stakeholders in various social campaigns that incorporate awareness about domestic violence, the helplines involved, and the legal provisions can be helpful. The MHE department of the National Institute of Mental Health and Neurosciences has already been doing novel work in the field of COVID-19 awareness using social media campaigns^3^. Social media is uniquely equipped to support this cause due to its high penetration and consumption. In certain countries such as France and Spain, pharmacies are being involved through media awareness, where asking for “Mask-19” is a code for domestic violence alert^4^.
- *Integration of social and public health systems:* Mental health promotion needs to be integrated into health communication at all levels of care. The grassroots community workers, general physicians, and nurses face the maximum caseload and thus need to be trained to deliver awareness about domestic violence (39). Telemedicine facilities are probably an asset in these situations for digital training and communication. Voices and lived experiences of the survivors matter and need to be included for peer support and training. Other stakeholders are the police, the justice system, social services, researchers, non-governmental organizations, and administrators.
- *Media–physician collaboration*: Mental health and public health experts need to be collaborating actively with all forms of print and digital media to debunk misinformation and help them educate the community about abuse prevention.
- *Victim care:* Various forms of adjustment disorders, stress reactions, and post-traumatic stress disorders are prevalent in abuse victims. Depression, anxiety, and suicidality are frequent accompaniments. MHE measures can be critical in helping them avail counseling and treatment facilities, fight the stigma, and preserving their autonomy and self-esteem. Gatekeeper training can help with suicide prevention.

RETRACTED

## Epilog

In the dark times, it is a shoulder, a hand, or an emotional response that one needs to feel heard and catered to. In the current scenario where one cannot have the face-to-face individual session, these services need to be provided to the vulnerable and needy populations through telephone, online, or other virtual methods for which the necessary pamphlets or leaflets could be prepared and circulated through social media methods as promotion of mental health and protection of human rights. Besides, civil society and non-governmental organizations will play a critical role in assisting. It is a collective responsibility, and all of us, irrespective of educational or socioeconomic background, can aid in the prevention of this social evil. The government can promote “domestic abuse prevention” as an “essential service,” which raises the bar of importance. The Indian Pandemic Act of 1897 unquestionably needs modification; incorporating the needs related to domestic violence might be worthy. Citizens of the country need to be sensitive to identify the earliest signs of abuse and report them to the necessary authorities. Legal and administrative provisions should be hassle-free to enable more reporting and assurance to the victims. The National Helplines by the Ministry of Health and Family Welfare, Government of India, can integrate child and women safety services to make it more comprehensive. Importantly, the marked gaps in research and data related to monitoring and implementing the interventions in domestic abuse need to be filled with systematic studies. Longitudinal studies throughout the pandemic, culturally sensitive modes of data collection, qualitative research exploring the lived experiences of survivors, and systematic reporting, as well as community surveillance, will add to understanding the dimensions of IPV during COVID-19. India is a fertile ground for the same, considering the increased prevalence of this social evil. The Non-Collegiate Women's Education Board records and anecdotal reporting need to be supplemented by systematic data, which are currently lacking from India. The authors call upon an urgent integrated and comprehensive public-mental health approach as a key to IPV prevention in India during the ongoing crisis and mental health education as an essential tool. The COVID-19 pandemic might be yet another opportunity for us to relook and evaluate the gaps in our prevention and care of domestic violence before it is past the point of no return. To conclude, in the words of Kofman and Garfin (6), indeed, in present times, “home is not always a haven”!

## Data Availability Statement

The original contributions presented in the study are included in the article/supplementary material, further inquiries can be directed to the corresponding author/s.

## Author Contributions

All authors were involved in conceptualization, literature review, and drafting the manuscript. The final version was read and approved by all authors.

## Conflict of Interest

The authors declare that the research was conducted in the absence of any commercial or financial relationships that could be construed as a potential conflict of interest.

RETRACTED

## Footnotes

^1^Available online at: https://www.un.org/en/un-coronavirus-communications-team/make-prevention-and-redress-violence-against-women-key-part (accessed October 5, 2020).

^2^Available online at: https://theprint.in/india/domestic-violence-top-crime-against-women-sedition-cases-doubled-in-2018-ncrb-data/347814/ (accessed October 5, 2020).

^3^Available online at: https://www.thehindu.com/news/national/karnataka/nimhans-pitches-in-to-help-shun-stigma-and-psychosocial-trauma/article31283585.ece (accessed October 5, 2020).

^4^Available online at: https://edition.cnn.com/2020/04/02/europe/domestic-violence-coronavirus-lockdown-intl/index.html (accessed October 5, 2020).
